The article "Effects of the Combination of Continuous Nursing Care and Breathing Exercises on Respiratory Function, Self-Efficacy, and Sleep Disorders in Patients with Lung Cancer Discharged from Hospital" was published in 2022. Journal: Contrast Media Mol Imaging.

# Effects of the Combination of Continuous Nursing Care and Breathing Exercises on Respiratory Function, Self-Efficacy, and Sleep Disorders in Patients with Lung Cancer Discharged from Hospital

**DOI:** 10.1155/2022/3807265

**Published:** 2022-07-31

**Authors:** Juan Du

**Affiliations:** Department of Respiratory and Critical Care Medicine, The First Affiliated Hospital Xi'an Jiao Tong University, Xi'an, China

## Abstract

The purpose of this study was to explore the effect of respiratory function and self-efficacy of patients with lung cancer after surgery by the combination of continuing nursing care and breathing exercises and to assess its clinical value in improving the quality of patients' sleep. 120 cases of lung cancer patients were divided into the control group (*n* = 60 cases) and the experimental group (*n* = 60 cases) randomly. The control group used conventional care methods for postoperative lung cancer patients, while the experimental group used continuous care combined with a respiratory exercise care model on the basis of conventional care, comparing the differences in the recovery of lung function, self-efficacy, sleep quality, incidence of sleep disorders, and other indicators between the two groups. The average indicator of recovery condition in patients of experimental groups FEV1 (L), FEV1% pred (%), and FEV1/FVC (%) was higher than patients in control groups with lower symptom scores and complication rates (*P* < 0.05). The self-efficacy score of patients in the experimental group was higher than that in the control group (*P* < 0.05) during sixty days of follow-up. The sleeping time of the experimental group was significantly shorter than that of the control group (*P* < 0.05) and the sleep time was longer than that of the control group (*P* < 0.05), but the incidence of sleep disorders and drug use rate were lower than that of the control group (*P* < 0.05) before discharge. Continuous nursing care combined with respiratory exercises can significantly accelerate the recovery of lung function and respiratory function reconstruction in patients with lung cancer after surgery, improve the self-efficacy score of patients, improve the sleep quality of patients, and be conducive to postoperative rehabilitation of patients.

## 1. Introduction

Lung cancer is a kind of malignant tumor which takes the first place of all those whose oncobiology has the characteristics of rapid progress, early dispersal transfer, and unfavorable clinic prognosis [1]. Owing to the promotion of low-dose CT screening of the chest and the application of neoadjuvant chemotherapy, more and more patients have access to radical treatment such as surgical resection; but at the same time, the perioperative care of lung cancer patients has become more demanding [2]. Perfect postoperative management is not only a necessary step to smoothly pass the operation period and comprehensively improve the long-term prognosis but also a basic requirement of the concept of accelerated rehabilitation surgery advocated in recent years. Sleep disorders are one of the most common maladaptive reactions in surgical inpatients and are a phenomenon of sleep-wake biorhythm alternation.

The article "Effects of the Combination of Continuous Nursing Care and Breathing Exercises on Respiratory Function, Self-Efficacy, and Sleep Disorders in Patients with Lung Cancer Discharged from Hospital" was published in 2022. Journal: Contrast Media Mol Imaging.

About 60%–90% of lung cancer patients have different degrees of sleep disturbance after surgery. The reasons for this are, in addition to factors inherent to surgery such as change in living environment, medical traumatic stress, and the influence of drains, it is also related to the disruption of gas exchange and hypoxemia due to the disruption of the anatomical and physiological structure of the lung by lung surgery [3]. Therefore, early and adequate breathing exercises are significantly important to the reconstruction of lung function, improvement of hypoxemia, and improvement of sleep quality. However, we discovered from clinic practice that the completeness of breathing exercise plans for patients discharged from the hospital is normally low, which is commonly related to the heavy beating exercise progress and low self-consciousness degree of patients [4]. The conventional nursing mode lacks continuity guidance and systematic follow-up after discharge and cannot meet the needs of postoperative respiratory exercise for patients with lung cancer at the present stage [5]. Continuous nursing care is a new nursing model advocated at the present stage, which is characterized by continuous and standardized nursing intervention for patients after discharge to comprehensively improve the long-term prognosis of patients. We reviewed the literature and found relatively few applications of continuous nursing care to lung cancer surgery. This study intends to explore the clinical nursing value of continuous nursing combined with respiratory exercise in improving respiratory function and sleep quality of patients after lung cancer surgery, in order to provide the nursing basis for the improvement of respiratory exercise and sleep quality of patients after lung cancer surgery.

## 2. Patients and Methods

### 2.1. Patients

120 cases of lung cancer patients with surgical indications received and cured by the First Affiliated Hospital of Xi'an Jiaotong University were adopted as study objects. The inclusive standard was as follows: definitive diagnosis: the patient was diagnosed with primary lung cancer by biopsy and bronchoscopy [6]; life expectancy was longer than 12 months; general surgical indications: within lung cancer stage II, no mediastinal lymph node metastasis; and clear mind, good cognitive function, rehabilitation, and exercise coordination qualified. The exclusive standard was as follows: complicated with primary lung diseases such as lung infection, active pulmonary tuberculosis, and severe COPD; patients with severe extrapulmonary systemic diseases and adverse systemic conditions; patients with previous chest and lung surgery; and incomplete medical history and lost follow-up. All of the study objects were divided into the control group (*n* = 60 cases) and the experimental group (*n* = 60 cases) randomly, and the two groups of patients' medical history and systemic condition are comparative (*P* > 0.05), as given in Table 1. The patients and their families gave informed consent, and the study protocol was reviewed and approved by the First Affiliated Hospital of Xi'an Jiaotong University Clinical Research Ethics Committee.

The article "Effects of the Combination of Continuous Nursing Care and Breathing Exercises on Respiratory Function, Self-Efficacy, and Sleep Disorders in Patients with Lung Cancer Discharged from Hospital" was published in 2022. Journal: Contrast Media Mol Imaging.

### 2.2. Study Methods

Conventional nursing methods after lung cancer surgery were adopted in the control group. (1) General breathing exercises in the hospital: we ordered patients to put their hands on their abdomen to give certain positive pressure and breathe in slowly and deeply. After the maximum deep inhalation, hold your breath for 5 seconds and then slowly exhale. Balloons can be blown to assist exercise for 15 minutes at a time, 3-4 times a day. (2) Medical pain management: we treated patients with conventional chest bandaging and fixation after surgery. The accompanying family member or the tube bed nurse could be asked to help fix the patient's chest when the patient coughs, which could reduce the pain caused by the incision or drainage tube displacement caused by posture changes. We guided patients to adopt an automatic epidural analgesia prescription. If necessary, patients followed the doctor's advice to use graded drug analgesia therapy. (3) Exercise and psychological care: we encouraged patients to get out of bed as soon as possible after the operation, pay attention to avoid pulling the drainage tube during the activity, and to first practice walking at the bedside and gradually increased the amount of exercise. We communicated with the patients frequently, learned about their psychological condition, and gave timely psychological counseling. In the experimental group, the continuous nursing combined with respiratory exercise nursing mode was adopted on the basis of routine nursing. (1) Guide before discharging from the hospital [7]: we set up a multidisciplinary continuous nursing care group for patients with lung cancer after surgery that consists of nursing staff, rehabilitation exercisers, psychological consultants, and patients' families and community respiratory rehabilitation personnel to create a continuous nursing file for each patient in the study group with the diagnosis and treatment process like age, course of disease, and surgical method well recorded, and the patient's information of family address and contact. We assessed the patient's existing respiratory function and pulmonary symptoms and assessed sleep quality and the risk of subsequent sleep disorders. We made an understanding of the family care capacity of each patient's family members. Care conditions were not ideal and other diseases were the focus of the group. Sleep disorders and some respiratory symptoms are often overlooked after discharge, so it was important to guide patients and their families to recognize symptoms. (2) Conduction of continuous nursing care [8]: we conducted continuous nursing care in the form of a questionnaire, made a clear understanding of time, purpose, and key points, communicated methods of each follow-up visit to make sure that the valuable current information of patients and the effect of rehabilitation exercise can be received on time, and provided guidance and assistance to patients if there are any discomforts or problems during the recovery period. As to patients with poor compliance, a one-to-one responsible system was adopted to closely follow the exercise outcome of each patient. According to the condition of patients to establish a multichannel continuity of care platform, such as the establishment of nailing discussion groups, did breathing exercises every day, and sleep intervention questionnaire collection and answering questions especially strengthen the respiratory exercise education, make treatment with in-depth understanding in patients with lower respiratory exercises after the operation, and the significance of improving patients' participation. Strengthen patients' ability to self-efficacy improvement and psychological crisis intervention and actively guide patients who were negative and pessimistic about the world and had no confidence in breathing exercise. (3) New breathing exercise nursing: breathing exercise during admission was the same as the control group, and rehabilitation exercise after discharge was simple and systematic breathing exercise, referring to the following steps [9]: calm breathing, vertical inhalation, forward exhalation; upper limbs lifted inspiratory, hands pressed abdomen expiratory; breathed in with your upper limbs flat and exhaled with your arms down; flat extended the upper limbs to inhale, press the abdomen with both the hands and exhale; patients were trained to breathe in, turn, and exhale; upper limb lift inhale; squat exhale; abdominal lip constriction breathing; and quiet breathing. Patients did it 3-4 sets daily.

The article "Effects of the Combination of Continuous Nursing Care and Breathing Exercises on Respiratory Function, Self-Efficacy, and Sleep Disorders in Patients with Lung Cancer Discharged from Hospital" was published in 2022. Journal: Contrast Media Mol Imaging.

### 2.3. Observation Target

Reconstruction condition of respiratory function [9]: the first second forced expiratory volume (FEV), the ratio of the first second forced expiratory volume to the expected value (FEV% PRED), and FEV/FVC were compared between the two groups after operation and 60 days after rehabilitation exercise. Data were measured at 60 days after intervention at the time of the patient's visit for review. Incidence of pulmonary symptoms and complications: revisionary modified lung cancer module MD Anderson Symptom Assessment Scale (MDASI) can conduct an assessment of patients' symptoms after surgery and 60 days later. Items included cough, sputum, hemoptysis, chest tightness, and weight loss, on a scale of 0–10, with 0 indicating symptoms disappearing and 10 indicating symptoms seriously affecting life. The incidence of pulmonary infection, atelectasis, and other complications was analyzed [10]. Improvement of self-efficacy and emotions: the modified version of the Nursing Care Self-Efficacy Scale (NURSES) was used to evaluate the patients' self-efficacy. The Hamilton depression scale (HAMD) and Hamilton anxiety scale (HAMA) were used to evaluate patients' depression and anxiety. The higher the score, the more serious the degree of depression or anxiety. Evaluation of sleep quality: the sleep quality of patients is measured by a self-made sleep quality questionnaire during hospitalization in our own hospital. The average time of falling asleep, sleeping time, incidence of sleep disorders, and frequency of sleep AIDS data are collected and counted before the patients are discharged from the hospital to evaluate the sleep quality of patients before and after nursing.

### 2.4. Statistical Analysis

Data of all patients are analyzed and handled by the Statistical Product and Service Solutions (SPSS) 24.00 (IBM, Armonk, NY, USA). Measurement data are expressed by ($\bar{x}\pm s$) and tested by *t*; enumeration data are tested by *χ*^2^. *P* < 0.05 is considered statistically significant.

## 3. Results

### 3.1. Systematic Conditions in the Two Groups of Patients

In this clinical study, a total of 120 patients with lung cancer who had the surgical opportunity were recruited and randomly divided into the control group and experimental group. Patients were followed up 60 days after being discharged from the hospital. The two groups were comparable in the aspects of age, gender composition, course of the disease, and surgical indicators (*P* > 0.06), as given in Table 1.

The article "Effects of the Combination of Continuous Nursing Care and Breathing Exercises on Respiratory Function, Self-Efficacy, and Sleep Disorders in Patients with Lung Cancer Discharged from Hospital" was published in 2022. Journal: Contrast Media Mol Imaging.

### 3.2. Breathing Function in the Two Groups of Patients

There was no difference in indexes of FEV1 (L), FEV1% PRED (%), and FEV1/FVC (%) lung function between the two groups after lung cancer surgery (*P* > 0.05). FEV1 (L), FEV1% pred (%), and FEV1/FVC (%) in the experimental group are higher than those in the control group (*P* < 0.05), as given in Table 2.

### 3.3. Incidence Rate of Respiratory System Symptoms and Complications in the Two Groups of Patients

There was no difference in the MDASI score of postoperative respiratory symptoms between the two groups (*P* > 0.05), while the score of the experimental group was significantly lower than that of the control group during the follow-up visit 60 days after surgery (*P* < 0.05), as given in Table 3.

### 3.4. Incidence Rate of Complications in the Two Groups of Patients

The complication incidence rate is significantly lower for patients in the experimental group than in the control group, as given in Table 4.

### 3.5. Comparison of Self-Efficacy and Depression and Anxiety Scores between the Two Groups of Patients

There are no differences in the Hamilton depression score, Hamilton depression and anxiety score, and self-efficacy between the two groups after surgery (*P* > 0.05), and 60 days after surgery, depression and anxiety scores of the experimental group are lower than those of the control group (*P* < 0.05) and the self-efficacy score is higher than that of the control group (*P* < 0.05), as given in Table 5. Before discharge from the hospital, the sleep time of the experimental group is obviously shorter than that of the control group (*P* < 0.05) and the sleep time is longer than that of the control group (*P* < 0.05), while the incidence of sleep disorders and drug use rate are lower than that of the control group (*P* < 0.05), as given in Table 6.

## 4. Discussion

Advances in clinical care have made radical treatment available to many patients with progressive lung cancer who would not otherwise have access to surgery [11] and have led to a significant increase in the number of patients hospitalized for lung cancer surgery, posing additional challenges to clinical care and perioperative care, of which treatment-related sleep disorders are a key concern for nursing staff. Among hospitalized patients with lung cancer, structural sleep disorders such as prolonged sleep time, sleep disruption, and early awakening are the most common. Long-term sleep disorders can make patients physically tired, reduce the intensity and efficiency of postoperative rehabilitation exercises, weaken patients' immune resistance, increase the risk of various postoperative infections, or lead to delayed wound healing. Patients with lung cancer are generally elderly and complicated with various organic cardiovascular diseases. Sleep disorders and hypoxemia may increase the possibility of cardiovascular events in patients. At the same time, sleep disorders can lead to depressed mood in patients, reduce their treatment compliance, reduce the quality of generation and self-cognitive efficacy of patients, and seriously threaten the prognosis of patients. After sleep improvement intervention for patients with lung cancer, it is found [12] that high-quality sleep can significantly improve the physical function and role cognition of patients with lung cancer and increase their response to treatment. Compared with general surgery, lung tissue resection had certain particularities, but there were few reports on the intervention of insomnia disorder in patients with lung cancer after surgery. The occurrence of postoperative insomnia disorder in patients with lung cancer is multifactored. Besides the inherent causes such as surgical stress and incision pain, it is also related to the pulmonary ventilation function and mediastinal cardiovascular hemodynamic disorder caused by thoracopulmonary surgery. Surgical stress and incision can be recovered in a few months, but cardiopulmonary ventilator-blood flow change is a long-term process with a very long adaptation stage [13]. Therefore, quality of life interventions, including sleep and respiratory function exercise, should be emphasized for patients undergoing lung cancer surgery.

The article "Effects of the Combination of Continuous Nursing Care and Breathing Exercises on Respiratory Function, Self-Efficacy, and Sleep Disorders in Patients with Lung Cancer Discharged from Hospital" was published in 2022. Journal: Contrast Media Mol Imaging.

The concept of continuous nursing care originated from chronic disease care and community health intervention to ensure coordination and continuity of healthcare services for patients in different medical and health places or in the same place with different levels of care [14]. At present, the mainstream mode of continuous nursing care in China includes three aspects: care arrangement, patient education, and service coordination. Lung cancer resection changes the anatomical and physiological environment of the patient's lung tissue, while the tissue incision may cause a localized injury stress response, which will affect the lung ventilation function of the patient, and in severe cases, may cause atelectasis. Effective respiratory exercise is of positive significance for rebuilding the patient's respiratory function and preventing complications. The existing respiratory function exercise is mainly to increase the front and back diameter of patients' thorax through regular breathing exercise and assist patients to maximize the expansion of lung capacity and improve respiratory muscle function. A malignant tumor is a chronic disease. Meanwhile, for patients with lung cancer after surgery, the change in respiratory function is lifelong, which also leads to the disorder of sleep rhythm, and its correction is a long-term process. The effectiveness of postoperative sleep intervention for patients with lung cancer depends on effective disease management after discharge [15]. The development of continuous nursing care mode enables patients with lung cancer to receive continuous and correct sleep intervention and respiratory exercise services in different healthcare settings. In China, postoperative lung cancer patients are discharged from the hospital to their home or communities, transfer of this phase is the content of the need to focus on nursing work, and continuity of care concept guide hospitals and community families in around the time of discharge in promoting breathing exercise, continuity, coordination of activities such as psychological care, and can realize smooth safe in patients with excessive, to improve the validity of the breathing exercise to improve the discharge end.

The article "Effects of the Combination of Continuous Nursing Care and Breathing Exercises on Respiratory Function, Self-Efficacy, and Sleep Disorders in Patients with Lung Cancer Discharged from Hospital" was published in 2022. Journal: Contrast Media Mol Imaging.

The continuous care model adopted in this study is a four-stage model carried out in China. The first is to make a comprehensive assessment of the patient's health status, family care ability, and available resources in the community before discharge. According to the situation of the patients, family, and community, individualized breathing exercise, psychological intervention, and sleep assistance plan and goal are made. Taking the individual differences of patients and their families into consideration, inviting primary caregivers to participate in the basic needs assessment and planning process at the beginning of the plan can identify the patients' sleep disorders and difficulties in breathing exercise. The second is effective hospital health education. Since the heterogeneity of lung cancer surgery is larger, the current state of the patients' health and rehabilitation goals are not the same. For the patient and family, people's health education effectively promotes the patient's breathing exercise tolerance and confidence, urging patients to complete their exercises with good quality, and is an effective measure to ease breathing disorders and sleep disorders. Psychological factors are more controllable factors in respiratory rehabilitation exercises and postoperative insomnia in lung cancer patients [16], so this should also be a key focus of continuing care. In recent years, due to the misplacement of media propaganda, lung cancer is a kind of cancer with high mortality and low treatment rate, which affects many patients. The vast majority of lung cancer patients have doubts about the benefit of treatment, so most patients will have anxiety and resistance to surgery and postoperative rehabilitation exercises and breathing exercises, with the most significant reaction at night. Therefore, in this study, relaxation exercises of conformal patients' own situations are adopted in the continuous care, such as progressive relaxation, meditative relaxation, and reflex muscle relaxation training, which have a good effect on reducing the postoperative body tension level of patients and alleviating their negative emotions. Nursing care after the discharge arrangement is the principal part. The continuity of care for patients in time on postoperative visit, appointment and booking arrangements, and the subsequent takeover of health care workers to communicate and to collect the complete patient information, so as to understand the patient's current self-efficacy, sleep quality, and breathing exercise effectiveness assessment, timely find patients' breathing exercise and exercise plan adjustment. However, related nursing work is often lacking in this aspect [17]. Researchers believe that the establishment of a multiperson continuous care team, especially to ensure that the team members include family members and community personnel, in order to achieve timely communication of the patient's situation, better carries out the continuity of care services related to respiratory exercise after lung cancer surgery. In this study, the incidence of sleep disorders and drug usage rate are lower than those in the control group (*P* < 0.05). However, due to the high threshold of the sleep quality evaluation, this study cannot carry out a strict evaluation of sleep quality of patients after discharge, or a more detailed return visit can be carried out jointly with community hospitals. At the follow-up visit 60 days after surgery, the lung function index of the experimental group is higher than that of the control group (*P* < 0.05), the symptom score and the complication rate are lower (*P* < 0.05), and the self-efficacy score is higher than that of the control group (*P* < 0.05). The reason lies in that same time of exercise, often with medium and low intensity load exercise, in order to increase pulmonary blood flow, conducive to pulmonary circulatory oxygenation. The current study still has some limitations. The sample size in this study is small and thus should be further validated by a further study with a larger sample size.

The article "Effects of the Combination of Continuous Nursing Care and Breathing Exercises on Respiratory Function, Self-Efficacy, and Sleep Disorders in Patients with Lung Cancer Discharged from Hospital" was published in 2022. Journal: Contrast Media Mol Imaging.

## 5. Conclusion

In conclusion, continuous nursing care combined with breathing function exercise improves the effectiveness and compliance of patients' postoperative rehabilitation effectively, heightens the self-efficacy of patients, and remarkably reduces the occurrence of various sleep disorders, which has a positive meaning for the reconstruction of respiratory function and physical rehabilitation of patients after operation.

## Figures and Tables

**Table 1:** Comparison of general conditions between the two groups.

Group	Number of subjects	Age (years)	Number of males (%)	Disease duration (months)	Procedure time (hours)	BMI (kg/m^2^)
Control group	60	65.23 ± 11.21	47 (73.33)	5.12 ± 3.44	4.12 ± 1.14	24.40 ± 3.11
Test group	60	65.21 ± 11.21	46 (76.66)	5.11 ± 3.54	4.12 ± 1.13	24.41 ± 3.21
*t*/*x*^2^		0.009	0.923	0.000	0.134	0.007
*P*		0.922	0.784	1.000	0.813	0.928

**Table 2:** Comparison of respiratory function between the two groups ($\bar{x}\pm s$).

Group	Number of subjects	FEV1 (L)		FEV1% pred (%)		FEV1/FVC (%)	
		Before surgery	60 days postoperative	Before surgery	60 days postoperative	Before surgery	60 dayspostoperative
Control group	60	1.39 ± 0.34	1.52 ± 0.36	54.82 ± 6.13	57.45 ± 2.46	60.54 ± 6.34	62.21 ± 1.82
Test group	60	1.37 ± 0.35	2.31 ± 0.22	55.18 ± 5.94	64.71 ± 2.44	60.21 ± 6.48	68.52 ± 1.94
*t*		0.348	15.889	0.358	17.779	0.309	20.128
*P*		0.729	0.000	0.721	0.000	0.758	0.000

**Table 3:** Comparison of MDASI scores between the two groups ($\bar{x}\pm s$).

Group	Number of subjects	Postoperative	60 dayspostoperative
Test group	60	26.77 ± 2.05	18.83 ± 1.37
Control group	60	27.13 ± 2.39	22.53 ± 1.83
*t*		0.639	8.863
*P*		0.526	<0.001

**Table 4:** Comparison of incidence rate of pulmonary complications between the two groups (*n* (%)).

Group	Number of subjects	Atelectasis	Lung infection	Local wound infection	Total occurrence
Test group	60	0 (0.00)	2 (3.33)	0 (0.00)	2 (3.33)
Control group	60	1 (1.67)	8 (13.33)	0 (0.00)	9 (15.00)
*X* ^2^					4.234
*P*					0.032

**Table 5:** Comparison of psychological status and self-efficacy between the two groups ($\bar{x}\pm s$, minutes).

Group	Number of subjects	HAMD		HAMA		Self-efficacy score	
		Postoperative	60 days postoperative	Postoperative	60 days postoperative	Postoperative	60 dayspostoperative
Test group	60	33.1 ± 3.1	19.5 ± 2.8	25.5 ± 4.4	12.5 ± 3.0	21.4 ± 4.3	29.6 ± 4.0
Control group	60	34.3 ± 3.1	24.0 ± 3.0	25.0 ± 3.6	17.3 ± 1.9	21.1 ± 2.4	24.5 ± 3.5
*t*		1.79	6.92	0.59	8.39	0.32	6.01
*P*		0.091	0.003	0.055	0.001	0.067	0.017

**Table 6:** Comparison of sleep between the two groups.

Group	Number of subjects	Time to fall asleep (hours)	Sleep duration (hours)	Incidence of sleep disorder (%)	Drug use rate (%)
Test group	60	1.02 ± 0.92	6.32 ± 2.11	49.45	23.45
Control group	60	1.53 ± 1.22	5.75 ± 2.77	69.33	39.43
*t*/*x*^2^		2.585	2.825	4.035	4.001
*P*		0.011	0.005	0.045	0.049

## Data Availability

The datasets used and analyzed during the current study are available from the corresponding author upon request.
